# Interleukin-1β-Induced Autophagy-Related Gene 5 Regulates Proliferation of Embryonic Stem Cell-Derived Odontoblastic Cells

**DOI:** 10.1371/journal.pone.0124542

**Published:** 2015-04-20

**Authors:** Nobuaki Ozeki, Naoko Hase, Taiki Hiyama, Hideyuki Yamaguchi, Rie Kawai, Ayami Kondo, Toru Matsumoto, Kazuhiko Nakata, Makio Mogi

**Affiliations:** 1 Department of Endodontics, School of Dentistry, Aichi Gakuin University, 2–11 Suemori-dori, Chikusa-ku, Nagoya, Aichi, 464–8651, Japan; 2 Department of Medicinal Biochemistry, School of Pharmacy, Aichi Gakuin University, 1–100 Kusumoto, Chikusa-ku, Nagoya, 464–8650, Japan; School of Medicine, University of Belgrade, SERBIA

## Abstract

We previously established a method for the differentiation of induced pluripotent stem cells and embryonic stem cells into α2 integrin-positive odontoblast-like cells. We also reported that Wnt5 in response to interleukin (IL)-1β induces matrix metalloproteinase (MMP)-3-regulated cell proliferation in these cells. Our findings suggest that MMP-3 plays a potentially unique physiological role in the generation of odontoblast-like cells under an inflammatory state. Here, we examined whether up-regulation of autophagy-related gene (Atg) 5 by IL-1β was mediated by Wnt5 signaling, thus leading to increased proliferation of odontoblast-like cells. IL-1β increased the mRNA and protein levels of Atg5, microtubule-associated protein 1 light chain (LC3, a mammalian homolog of yeast Atg8) and Atg12. Treatment with siRNAs against Atg5, but not LC3 and Atg12, suppressed the IL-1β-induced increase in MMP-3 expression and cell proliferation. Our siRNA analyses combined with western blot analysis revealed a unique sequential cascade involving Atg5, Wnt5a and MMP-3, which resulted in the potent increase in odontoblastic cell proliferation. These results demonstrate the unique involvement of Atg5 in IL-1β-induced proliferation of embryonic stem cell-derived odontoblast-like cells.

## Introduction

Macroautophagy (hereafter referred to as autophagy) is an evolutionarily conserved ubiquitous cellular process [1]. Autophagy has important functions in resistance to starvation, maintenance of cellular functions, growth control, and removal of anomalous cellular components that accumulate during cell aging [2–4]. Among the approximately 30 autophagy-related genes (Atgs) identified to date, Atg5, Atg12 and microtubule-associated protein 1 light chain (LC3, a mammalian homolog of yeast Atg8), are specifically involved in two ubiquitin-like protein conjugation systems (Atg5-Atg12 and LC3-phosphatidylethanolamine). Both systems are responsible for the sequestration process of autophagy [5]. Of note, recent studies have found that autophagy affects innate and adaptive immunity, inflammation and apoptosis, thereby potentially influencing their corresponding pathological processes [6–8]. Compelling evidence indicates that autophagy participates in the pathogenesis of diverse neurodegenerative diseases, cancer and inflammatory diseases, including arthritis and periodontitis [9–12]. However, the physiological function of Atgs on bone-related cells, especially odontoblasts, has not been well defined.

The dental pulp is a highly innervated tissue with sensory axons mainly distributed in the dentin-pulp complex. Dental pulp consists predominantly of odontoblasts with smaller populations of fibroblasts, as well as blood vessels [13–15]. The early inflammatory response to caries is characterized by focal accumulation of chronic inflammatory cells, which is mediated initially by odontoblasts and later by dendritic cells. As the most peripheral cells in the pulp, odontoblasts are positioned to encounter foreign antigens first and initiate the innate immune response [16,17]. Once the toll-like receptor family in odontoblasts is stimulated by a pathogen, proinflammatory cytokines, chemokines, and antimicrobial peptides are secreted by the odontoblasts, resulting in recruitment and stimulation of immune effector cells as well as direct bacterial killing [18]. Therefore, odontoblasts may represent a new target for pulpitis treatment. However, obtaining sufficient numbers of purified odontoblasts is challenging, which has hampered research into odontoblasts following induction of inflammation. Thus, we have performed experiments using purified odontoblast-like cells derived from induced pluripotent stem (iPS) cells [19] and embryonic stem (ES) cells [20]. These odontoblast-like cells are excellent *in vitro* models to examine the mechanisms of wound healing in diseased areas such as inflammatory sites during dental caries or inflamed dental pulp.

Matrix metalloproteinases (MMPs) are a family of calcium- and zinc-dependent extracellular matrix-degrading enzymes that participate in both physiological and pathophysiological processes. Our previous studies reported that MMP-3 accelerates wound healing following dental pulp injury [21,22]. We have also reported that the proinflammatory cytokine interleukin (IL)-1β induces an increase in Wnt5 signaling, leading to MMP-3 expression and promotion of cell proliferation [23]. This signaling cascade appears to be in the order of IL-1β→Wnt5→Lrp5/Fzd9→MMP-3, and is intimately involved in cell proliferation in stem cell-derived odontoblast-like cells. This observation indicates that MMP-3 may instead be involved in extracellular matrix degradation and subsequent morphogenesis, wound repair [21,22] and angiogenesis [21,22,24], within the inflamed tissue. However, no study has focused on Atgs in cell proliferation, especially odontoblastic cell proliferation. Therefore, further studies are required to completely understand its intracellular role in odontoblasts.

Here, we examined whether Atg signaling is associated with the expression of MMP-3 during odontoblast proliferation that may occur in inflamed dental pulp. Our study of mouse iPS and ES cell-derived odontoblast-like cells aimed to delineate the degree of involvement of Atg5 in the expression of MMP-3, and the factors that regulate this process. We show for the first time that Atg5 up-regulates MMP-3 expression with an increase in Wnt5 signaling in odontoblast-like cells, leading to enhanced cell proliferation.

## Materials and Methods

### Cell Culture

The mouse iPS cell line iPS-MEF-Ng-20D-17 [25] was a kind gift from Prof. Shinya Yamanaka (Center for iPS Cell Research and Application, Kyoto University, Kyoto, Japan) and was maintained as described previously [25,26]. Similarly, the mouse ES cell line E14Tg2a [27] was a kind gift from Dr. Randall H. Kramer (University of California, San Francisco, CA, USA) and was maintained as described previously [28]. B6G-2 ES cells were purchased from the Riken Cell Bank (Ibaraki, Japan) and were maintained as described previously [29]. Because B6G-2 cells require a feeder cell layer and E14Tg2a cells do not, these cell lines were used for comparison. Rat odontoblast-like KN-3 cells [30] were kindly provided by Dr. Chiaki Kitamura (Kyushu Dental College, Kitakyushu, Japan), were maintained as described previously [30] and used as an authentic control. Purified odontoblast-like cells derived from both ES cells [20] and iPS cells [19] were prepared as reported previously. In brief, monoclonal anti-α2 integrin antibody is known to potently suppress the expression of odontoblastic markers in these culture systems. We have previously confirmed that α2 integrin expression in ES cells triggers their differentiation into odontoblast-like cells [20]. The proportion of α2 integrin-positive cells in the total population of differentiated odontoblast-like cells is a measure of the purity of ES cell-derived odontoblast-like cell preparations. Flow cytometric analysis estimated the proportion of odontoblast-like cells to be 98.54±0.45% (iPS cell derived; *n* = 3), 98.24±0.68% (B6G-2 cell derived; *n* = 3) and 98.54±0.47% (E14Tg2a cell derived; *n* = 3). Up to day 21 of culture, these differentiated cells displayed odontoblast-like physiological characteristics including calcification activity and alkaline phosphatase activation.

### Cell proliferation assay and microscopic analysis

Cell proliferation was evaluated by the BrdU-cell proliferation enzyme-linked immunoabsorbent assay (ELISA; Roche Applied Science, Mannheim, Germany) as described previously [31,32]. The cells were seeded into 96-well culture plates at a density of 1×10^4^ cells/well. Cell proliferation was also evaluated visually under a BZ-9000 microscope (Keyence, Osaka, Japan) using the BrdU Immunohistochemistry Kit (Abcam, Cambridge, UK) according to the manufacturer’s instructions.

### Determination of apoptotic cell death

Apoptosis was evaluated visually under the BZ-9000 microscope using an APOPercentage Apoptosis Assay Kit (Funakoshi Co., Ltd., Tokyo, Japan) [33].

### Real-time quantitative polymerase chain reaction (qPCR) analysis

Real-time qPCR was performed in triplicate in 96-well optical microtiter plates with ~25 ng RNA, 0.25 μL Quantitect RT Mix (Qiagen, Valencia, CA, USA), 1.25 μL of 20× Primer/Probe Mix, and 12.5 μL Mastermix (Qiagen Quantitect RT-PCR kit) in a 25 μL reaction volume. The following primer/probe sets (Assays-On-Demand, Applied Biosystems, CA, USA) were used: mouse Atg5, Mm00504340_m1; mouse Map1lc3a (LC3), Mm00458725_g1; mouse Atg12, Mm00503201_m1; mouse Wnt5a, Mm00437347_m1; mouse MMP-3, Mm00440295_m1; rat Atg5, Rn01767063_m1; rat Map1lc3a (LC3), Rn00458724_g1; rat Atg12, Rn1491906_g1.

Standards and samples were mixed with the PCR reagents, loaded into the 96-well microtiter plate and sealed with optical film (Applied Biosystems). PCR cycling conditions were 30 min at 50°C, 15 min at 95°C, and then 40 cycles of 15 s at 94°C/60 s at 60°C. A standard curve was used for relative quantitation of gene expression. Glyceraldehyde-3-phosphate dehydrogenase (GAPDH) and 18S rRNA were employed as housekeeping genes for normalization of the amount of total RNA in each sample. The amounts of target and endogenous reference mRNA were then determined from the appropriate standard curve. The amount of target mRNA was then divided by the amount of endogenous reference mRNA to obtain a normalized target value. *Ct* (threshold cycle) values for target and housekeeping genes were extrapolated from the standard curve to produce an arbitrary value of expression, the ratio of which (target/housekeeping gene) within each sample was plotted as the relative mRNA expression level.

### Western blot analysis

Atg5, Wnt5a and MMP-3 protein levels in cell lysates were determined by western blot analysis. Cells were cultured for 24 h with or without IL-1β (Prepro Tech, Rocky Hill, NJ, USA), lysed and then protein samples were separated on 12% sodium dodecyl sulfate polyacrylamide gels. Western blot analysis was performed using anti-Atg5, anti-LC3, anti-Atg12, anti-Wnt5a, anti-MMP-3, and anti-β-tubulin polyclonal antibodies (sc-8667, sc-398822, sc-68884, sc-365370, sc-6839, and sc-9935, respectively; Santa Cruz Biotechnology Inc., Santa Cruz, CA, USA). The anti-Atg5 and anti-MMP-3 antibodies showed no significant cross-reactivity with other Atgs or MMPs, respectively (data not shown). Visualization and quantification of blotted protein bands were performed with Multi Gauge-Ver3.X software (Fujifilm).

### Measurement of MMP-3 activity

The protocol for measurement of MMP-3 activity has been described previously [34] based on a commercially available MMP-3 activity assay kit (SensoLyte 520 MMP-3 Assay Kit; AnaSpec, San Jose, CA, USA). Briefly, prior to detection, MMP-3 was immunoprecipitated from the culture medium using a goat anti-MMP-3 polyclonal antibody (sc-6839, Santa Cruz Biotechnology Inc.) and protein A/G-agarose for 6 h at 4°C. After centrifugation, the agarose pellets were suspended in MMP-3 assay buffer containing the MMP-3 substrate (5-FAM-Arg-Pro-Lys-Pro-Val-Glu-Nva-Trp-Arg-Lys-QXL 520-NH_2_ fluorescence resonance energy transfer peptide [35]), which was supplied in the assay kit. MMP-3 activity was then determined according to the manufacturer’s instructions.

### Silencing of Atg5, Wnt5a, and MMP-3 genes by siRNA transfection

Atg5, Wnt5a and MMP-3 siRNAs for gene silencing were acquired commercially (sc-41446, sc-41113 and sc-37265, respectively; Santa Cruz Biotechnology Inc.) and were transfected into cultured cells using an siRNA reagent system (Santa Cruz Biotechnology Inc.) according to the manufacturer’s protocol. GAPDH siRNA and control siRNA (Thermo Scientific, Lafayette, CO, USA) with no known homogeny for any vertebrate sequence were used as positive and negative controls, respectively.

### Statistical analysis

Data are shown as the means ± standard deviation (SD) of four to six independent experiments. Statistical significance was assessed using the Mann–Whitney U-test. A value of *P* < 0.05 was considered as statistically significant.

## Results

### IL-1β-mediated induction of Atg5 mRNA and protein expression

The two stem cell-derived odontoblast-like cell lines and KN-3 cells were cultured in the presence of four concentrations of IL-1β (0, 0.25, 2.5, and 25 ng/mL). Induction of Atg5 mRNA and protein was assessed by qPCR (Fig 1A–1D) and western blot analysis (Fig 1E–1H), respectively. The mRNA and protein levels of Atg5 were increased by IL-1β at 0.25 and 2.5 ng/mL, but not 25 ng/mL.

**Fig 1:** IL-1β-induced expression of Atg5 mRNA and protein in odontoblast-like cells. Two stem cell-derived odontoblast-like cell lines and an odontoblast cell line (KN-3) were treated with IL-1β (0, 0.25, 2.5, and 25 ng/mL). (A–D) qPCR analysis of Atg5 mRNA expression relative to the control (18S rRNA). Data are the means ± SD of four independent experiments. **P < 0.01. (E–H) Western blot analysis of Atg5 and β-tubulin protein levels following stimulation with IL-1β. Representative blots of three independent experiments are shown.

It is known that bone-associated cells express other Atgs such as LC3 and Atg12 [36,37]. To assess whether induction of LC3 and Atg12 by IL-1β is a specific response in stem cell-derived odontoblast-like cells, we evaluated the expression of these genes following treatment with the same concentrations of IL-1β (0, 0.25, 2.5 and 25 ng/mL). We found that the mRNA and protein levels of LC3 and Atg12 were also increased by IL-1β at 0.25 and 2.5 ng/mL, but not 25 ng/mL (Figs 2 and 3).

**Fig 2:** IL-1β-induced expression of LC3 mRNA and protein in odontoblast-like cells. Two stem cell-derived odontoblast-like cell lines and an odontoblast cell line (KN-3) were treated with IL-1β (0, 0.25, 2.5, and 25 ng/mL). (A–D) qPCR analysis of LC3 mRNA expression relative to the control (18S rRNA). Data are the means ± SD of four independent experiments. **P < 0.01. (E–H) Western blot analysis of LC3 and β-tubulin protein levels following stimulation with IL-1β. Representative blots of three independent experiments are shown.

**Fig 3:** IL-1β-induced expression of Atg12 mRNA and protein in odontoblast-like cells. Two stem cell-derived odontoblast-like cell lines and an odontoblast cell line (KN-3) were treated with IL-1β (0, 0.25, 2.5, and 25 ng/mL). (A–D) qPCR analysis of Atg12 mRNA expression relative to the control (18S rRNA). Data are the means ± SD of four independent experiments. **P < 0.01. (E–H) Western blot analysis of Atg12 and β-tubulin protein levels following stimulation with IL-1β. Representative blots of three independent experiments are shown.

### Effect of Atg5 siRNA on IL-1β-induced MMP-3 expression and cell proliferation

Subsequent experiments used ES cell-derived cells (E14Tg2a) with rat KN3 cells as authentic standard odontoblast-like cells. We next employed specific siRNAs to determine whether the effects of IL-1β stimulation were specifically mediated by Atg5, LC3 or Atg12. Cells were transfected with Atg5, LC3 and Atg12 siRNAs, or a control siRNA, and were then stimulated with IL-1β as described above. These siRNAs did not affect the expression of the internal control (*GAPDH*) after transfection. MMP-3 mRNA was expressed only in cells transfected with control siRNA with no apparent expression in cells transfected with only the Atg5 siRNA (Fig 4A). The lack of an effect by the negative control siRNA confirmed that these IL-1β-stimulated effects were specifically mediated by Atg5. However, LC3 and Atg12 siRNAs had no effect on the expression of MMP-3, suggesting that only Atg5 is associated with IL-1β-induced MMP-3 expression in these cells (Figs 5A and 6A). Western blot analysis of Atg5, Wnt5a and MMP-3 proteins confirmed efficient silencing of the Atg5 gene (Fig 4A, right row). siRNA transfection had no effect on the expression of β-tubulin (the loading control). Atg5 siRNA caused potent suppression of Wnt5a and MMP-3 induction, indicating that Atg5, Wnt5a and MMP-3 act in similar signaling pathways, and Atg5 is upstream of Wnt5a and MMP-3 in the signaling cascade.

**Fig 4:** Effect of Atg5 siRNA on IL-1β-induced MMP-3 activity and cell proliferation. (A) E14Tg2a ES cell-derived odontoblast-like cells were transfected with Atg5 siRNA for 24 h and treated with IL-1β (0, 0.25, 2.5 and 25 ng/mL) for either 12 h (grey bars) or 24 h (black bars), prior to carrying out an MMP-3 activity assay (left) and western blotting for Atg5, Wnt5a and MMP-3 (right). (B) Results of the BrdU-cell proliferation ELISA (for cell proliferation; graphs), BrdU Immunohistochemistry Kit (for cell proliferation; images, upper row), and APOPercentage Apoptosis Assay kit (for apoptosis; images, lower row) are shown. β-Tubulin was used as a housekeeping protein in western blots. **P < 0.01 *vs*. control; ^##^ *P* < 0.01 *vs*. control siRNA; ^†^ *P* < 0.01, as indicated by the bracket. The BrdU ELISA kit stains the nuclei of proliferating cells dark brown. Accumulation of dye (pink-purple) denotes apoptosis in the APOPercentage kit. Images are representative of at least three independent experiments. Scale bars = 100 μm.

**Fig 5:** Effect of LC3 siRNA on IL-1β-induced MMP-3 activity and cell proliferation. (A) E14Tg2a ES cell-derived odontoblast-like cells were transfected with LC3 siRNA for 24 h and treated with IL-1β (0, 0.25, 2.5 and 25 ng/mL) for either 12 h (grey bars) or 24 h (black bars), prior to carrying out an MMP-3 activity assay (left) and western blotting for LC3, Wnt5a and MMP-3 (right). (B) Results of the BrdU-cell proliferation ELISA (for cell proliferation; graphs), BrdU Immunohistochemistry Kit (for cell proliferation; images, upper row), and APOPercentage Apoptosis Assay Kit (for apoptosis; images, lower row) are shown. β-tubulin was used as a housekeeping protein in western blots. **P < 0.01 *vs*. control; ^##^ *P* < 0.01 *vs*. control siRNA; ^†^ *P* < 0.01, as indicated by the bracket. The BrdU ELISA kit stains the nuclei of proliferating cells dark brown. Accumulation of dye (pink-purple) denotes apoptosis in the APOPercentage kit. Images are representative of at least three independent experiments. Scale bars = 100 μm.

**Fig 6:** Effect of Atg12 siRNA on IL-1β-induced MMP-3 activity and cell proliferation. (A) E14Tg2a ES cell-derived odontoblast-like cells were transfected with Atg12 siRNA for 24 h and treated with IL-1β (0, 0.25, 2.5 and 25 ng/mL) for either 12 h (grey bars) or 24 h (black bars), prior to carrying out an MMP-3 activity assay (left) and western blotting for Atg12, Wnt5a and MMP-3 (right). (B) BrdU-cell proliferation ELISA (for cell proliferation; graphs), BrdU Immunohistochemistry Kit (for cell proliferation; images, upper row), and APOPercentage Apoptosis Assay Kit (for apoptosis; images, lower row). β-tubulin was used as a housekeeping protein in western blots. **P < 0.01 *vs*. control; ^##^ *P* < 0.01 *vs*. control siRNA; ^†^ *P* < 0.01, as indicated by the bracket. The BrdU ELISA kit stains the nuclei of proliferating cells dark brown. Accumulation of dye (pink-purple) denotes apoptosis in the APOPercentage kit. Images are representative of at least three independent experiments. Scale bars = 100 μm.

Under identical culture conditions, we tested the effect of Atg5 siRNA on IL-1β-induced changes in cell proliferation. Compared with untransfected and control siRNA-transfected cells, Atg5 silencing in IL-1β-stimulated odontoblast-like cells resulted in a considerable decrease in the number of proliferating cells (*P* < 0.01; Fig 4B). The reduction in the proliferative potential was estimated to be ~95%. These results were confirmed by microscopic analysis of cell proliferation and apoptosis (Fig 4B). Under similar conditions, LC3 and Atg12 siRNAs had no effect on cell proliferation (Figs 5B and 6B).

### Evaluation of the expression order during IL-1β-induced cell proliferation by siRNA silencing

Using several specific siRNAs, we examined the sequential order of Atg5, Wnt5 and MMP-3 expression in odontoblast-like cells by qPCR and western blot analysis (Fig 7A–7F). IL-1β-induced expression of Atg5 was only inhibited by Atg5 siRNA (Fig 7), whereas Wnt5a expression was inhibited by both Wnt5a and Atg5 siRNAs (Fig 7). Furthermore, IL-1β-induced MMP-3 expression was inhibited by Atg5, Wnt5a and MMP-3 siRNAs (Fig 7). Similar results were obtained from western blot analysis (Fig 7). Thus, taken together with the above data, this signaling cascade appears to be IL-1β→Atg5→Wnt5a→MMP-3 and is intimately involved in the proliferation of stem cell-derived odontoblast-like cells.

**Fig 7:** Determination of the signaling sequence using specific siRNAs. (A–F) Cells were incubated in serum-free medium for 24 h and then treated with IL-1β (0, 0.25, 2.5 and 25 ng/mL) and Atg5, Wnt5a, or MMP-3 siRNAs. mRNA expression levels of Atg5, Wnt5a and MMP-3 relative to the control (18S rRNA) were determined by qPCR and western blotting for LC3, Atg5, Wnt5a, and MMP-3 (lower row). β-tubulin was used as a housekeeping protein in western blots. **P < 0.01 *vs*. control; ^##^ *P* < 0.01 *vs*. control siRNA; ^†^ *P* < 0.01, as indicated by the bracket.

## Discussion

We have previously demonstrated that the proinflammatory cytokine IL-1β induces an increase in Wnt5 signaling, leading to MMP-3 expression, promotion of cell proliferation, and suppression of apoptosis in odontoblast-like cells and immortalized KN-3 cells [23]. Although other associated cells express additional MMPs, such as MMP-1, MMP-2, MMP-9, and MMP-13 [38–40], we found no significant increase in their expression levels in our odontoblast-like cells (data not shown).

Although the upstream molecules of Wnt5 signaling are unknown, we demonstrated that IL-1β was found to stimulate Atg5 expression and the Wnt5 signaling cascade, resulting in MMP-3 activation and up-regulation of odontoblast-like cell proliferation at first. This observation may represent a novel physiological function of Atg5 and might be physiologically relevant in counteracting the effects of inflammation induced by IL-1β.

Our data highlight four main points. First, this is the first study to use a specific siRNA targeting Atg5 to show the mechanism of IL-1β-induced proliferation in mouse ES cell-derived odontoblast-like cells. The lack of such a previous study is primarily because of the difficulty in generating sufficient numbers of odontoblast-like cells. No study has investigated the effect of MMP-3 silencing on cell proliferation in these cells, except for our previous reports [34,41]. While the use of human ES cells is ethically controversial and clinical treatments employing these cells are likely some way from realization [42], the advancement of our basic knowledge with regard to mouse ES cell-derived odontoblastic cells is nevertheless highly important. Because only single siRNA's are used to knock down specific genes, leaving open the possibility of off-target effects, additional supporting experiments might be needed in the near-future.

Second, Atg5, Atg12 and LC3, as mammalian homologs of yeast Atg8, are specifically involved in two ubiquitin-like protein conjugation systems (Atg5-Atg12 and LC3-phosphatidylethanolamine) that are responsible for the sequestration process of autophagy [5]. However, Atg5 was not associated with Atg12 in IL-1β-induced proliferation of odontoblastic cells (Fig 6). LC3 and Atg12 siRNAs had no effect on the expression of MMP-3 and cell proliferation (Figs 4–6). Therefore, we demonstrated a unique physiological significance of Atg5 in these cells.

Third, although it is known that the Wnt5 signaling pathway is involved in osteoblastic cell differentiation and apoptosis [43,44], we demonstrated that Wnt5a is the key factor in the proliferation of odontoblast-like cells as reported previously [23]. Because Atg5 is upstream of Wnt5, it is likely that Atg5 is the most important factor in the Wnt5-signaling pathway. It might be physiologically relevant in counteracting the effects of inflammation induced by IL-1β.

Finally, our most striking finding is that IL-1β-induced Atg5 and increased Wnt5 signaling, leading to MMP-3 expression, promotion of cell proliferation and suppression of apoptosis. *In vitro*, this activity might be associated with an anti-inflammatory effect in odontoblast-like cells. Because this signaling cascade appears to be IL-1β→Atg5→Wnt5a→MMP-3, Atg5 plays an important role in IL-1β-induced cell proliferation at a relatively early step in the signaling cascade. As shown in Fig 4, the combined weak inflammatory state induced by IL-1β and Atg5 siRNA resulted in potent suppression of cell proliferation, suggesting that Atg5 expression might be a key determinant for cell survival.

Because Atg proteins Atg5, Atg12, and LC3 are required for basal autophagy, it is likely that these proteins are constitutively expressed in all cell types. However, we found no basal protein expression of Atg5, Atg12, or LC3 in odontoblasts. It remains to be determined whether this phenomenon is specific to odontoblasts.

Our results demonstrate that different IL-1β concentrations exert opposing effects on cell proliferation in ES cell-derived odontoblast-like cells. As shown in Fig 4, IL-1β concentrations of 25 ng/mL, together with Atg5 siRNA transfection, resulted in apoptosis and a decrease in cell proliferation and MMP-3 expression. However, slightly lower concentrations (0.25 and 2.5 ng/mL) resulted in enhanced cell proliferation. We concluded that at low levels of IL-1β (for example during the early stages of inflammation), Atg5, Wnt5a and MMP-3 contribute to tissue healing during odontoblast inflammation. However, the physiological significance of this cascade and the underlying mechanism, especially for the basis for Atg actions, remains to be elucidated. Recently, we established conditions for efficient conversion of human muscle stem cells to an odontoblast lineage [42], which circumvents many of the ethical issues of human ES cells. We will use these cells to revisit our previous and current studies of mouse cells to determine the extent to which our findings are relevant to humans.

It is known that odontoblasts are long-lived postmitotic cells with an autophagic activity as an essential mechanism for maintenance and cell survival [13]. Because we found that Atg5 expression is involved in the MMP-3 signaling cascade, the autophagy protein Atg5 has additional roles in odontoblast-like cell proliferation. It is currently unknown whether this function is specific and/or limited to odontoblasts.

In summary, we have demonstrated that Atg5 responds to IL-1β by up-regulation of MMP-3 expression via the Wnt5 signaling pathway in mouse ES cell-derived odontoblast-like cells. This pathway leads to an increase in the proliferation of odontoblastic cells. These results provide new insights into the role of Atg5 in odontoblasts and may have relevance for our understanding of and ability to improve wound healing following dental pulp injury.
